The article "Comparison of the Value of Conventional Ultrasound and Contrast-Enhanced Ultrasound-Guided Puncture Biopsy in Different Sizes of Peripheral Pulmonary Lesions" was published in 2022. Journal: Contrast Media Mol Imaging.

# Comparison of the Value of Conventional Ultrasound and Contrast-Enhanced Ultrasound-Guided Puncture Biopsy in Different Sizes of Peripheral Pulmonary Lesions

**DOI:** 10.1155/2022/6425145

**Published:** 2022-05-09

**Authors:** Qi-Qin You, Shi-Yi Peng, Zhi-Ying Zhou, Xing-Li Tan, Xian-Sheng Miao

**Affiliations:** Department of Medical Ultrasound, Qingpu Brance of Zhongshan Hospital, Fudan University School of Medicine, No. 1158 East Park Road, Shanghai 201700, China

## Abstract

**Objective:**

To compare the clinical value of contrast-enhanced ultrasound and conventional ultrasound-guided puncture biopsy in peripulmonary lesions of different sizes.

**Materials and Methods:**

110 patients with peripulmonary lesions were randomly divided into two groups: the conventional ultrasound-guided group and the contrast-enhanced ultrasound-guided group. The lesions in the two groups were further divided into two groups according to the size of the lesions, and the tissues taken after puncture biopsy were sent for pathological examination. The pathological results were compared with the postoperative pathological results and other examination results, and the complications were recorded at the same time.

**Results:**

In the conventional ultrasound group, the success rate of single puncture was 72.7% and the success rate of puncture was 80.0%; in the contrast group, the success rate of single puncture was 90.9% and the success rate of puncture was 94.6%. The difference between the two groups was statistically significant. There was no significant difference in needle bleeding and pneumothorax between the two groups. In the <30 mm group, there was no significant difference in the success rate of single puncture and the success rate of puncture between the two groups according to the size of the lesions. In the ≥30 mm group, the success rate of single puncture (97.1%) and puncture success rate (97.1%) in the contrast guidance group were higher than those in the conventional ultrasound guidance group (70.3%, 78.4%) and the difference was statistically significant (*p* < 0.05).

**Conclusion:**

Compared with conventional ultrasound, for peripheral pulmonary lesions guided by contrast-enhanced ultrasonography, especially when the maximum diameter of the lesion is ≥ 30 mm, needle biopsy has better guiding significance; for peripheral lung lesions with a maximum diameter of <30 mm, contrast-enhanced ultrasonography is compared with conventional ultrasound guidance. The puncture success rate was not significantly different.

## 1. Introduction

Percutaneous lung biopsy is often used to obtain pathological diagnosis of peripheral pulmonary lesions (PPLs) to guide clinical treatment. Because the peripheral lung lesions are close to the pleura, the application of ultrasound makes it easy to display the lesions and ultrasound has the advantages of real-time visualization, simplicity, and freedom from ionizing radiation. Therefore, ultrasound is generally used clinically to guide the needle biopsy of peripheral lung lesions [1–3]. The key to the success of puncture biopsy is whether effective lesions can be obtained, but for lesions of different sizes, the probability of liquefaction and necrosis increases with the increase in lesions. If the tissue is necrotic, it will lead to the failure of puncture biopsy. Ultrasonic contrast, also known as acoustic contrast, is a technique that uses a contrast agent to enhance the backscattered echoes and significantly improves the resolution, sensitivity, and specificity of ultrasound diagnosis. With the improvement of instrument performance and the emergence of new acoustic contrast agents, CEUS can effectively enhance the two-dimensional ultrasound images and blood flow Doppler signals of the myocardium, liver, kidney, brain, and other solid organs and reflect and observe normal tissues and lesions. The blood perfusion of tissues has become a very important and promising development direction of ultrasound diagnosis. The new generation of ultrasound contrast agent can truly reflect the distribution of blood supply in the lesions, and it is easy to distinguish between effective and necrotic lesions, which is of guiding significance in lung biopsy [4–7]. The purpose of this study was to compare the accuracy of conventional ultrasound and contrast-enhanced ultrasound-guided needle biopsy in the diagnosis of peripheral pulmonary lesions and the incidence of complications and evaluate the application value of two methods in the guidance of needle biopsy of peripheral lung lesions.

## 2. Materials and Methods

### 2.1. Research Object

The subjects were selected from our hospital from January 2016 to March 2021. CT examination was performed, and it was diagnosed as peripheral pulmonary disease. Routine ultrasound or contrast-enhanced ultrasound-guided lung biopsy was performed, and cases confirmed by operation, pathology, or clinical follow-up results were obtained. Inclusion criteria were as follows: peripheral pulmonary lesions revealed by ultrasound. Exclusion criteria were as follows: (1) ultrasound that cannot clearly display lesions; (2) those with severe cardiopulmonary insufficiency; (3) patients with aortic aneurysm and pulmonary hypertension; (4) patients with bleeding tendency; (5) people with mental disorders; (6) people with severe cough; (7) patients with contrast agent allergy. After screening, 110 cases were enrolled in the group, including 73 males and 37 females. The age ranged from 20 to 90 years old, and the average age was (68.2 ± 13.6) years. Locations of lung lesions included 80 cases in middle and upper lobes and 30 cases in lower lobes. The maximum diameter of PPLs was the statistical index, the minimum was 19 mm, and the maximum was 137 mm. The average diameter of the lesion was (48.2 ± 24.6) mm. The cases were grouped and analyzed as follows.

Fifty-five patients in the conventional ultrasound group (conventional ultrasound-guided percutaneous lung biopsy) were further divided into <30 mm group of 18 cases and ≥30 mm group of 37 cases, according to the maximum diameter of the lesion (30 mm); fifty-five patients in the ultrasound contrast group (contrast-enhanced ultrasound followed by percutaneous lung biopsy under the guidance of ultrasound) were further divided into <30 mm group (*n* = 20) and ≥30 mm group (*n* = 35) according to the maximum diameter of the lesion (30 mm).

### 2.2. Instruments and Methods

The instrument used was the Yum Mylab Twice eHD Color Doppler ultrasound diagnostic instrument, and the instrument was equipped with corresponding ultrasound contrast software. The probe frequency was 3.5∼5.0 MHz. The biopsy device from American BARD was used, equipped with an 18G biopsy needle. The needle length was 20 cm, and the ejection distance was 22 mm.

#### 2.2.1. Preoperative Preparation

Preoperative routine examination obtained blood routine, serological and coagulation functions, and so on. A conventional ultrasound examination was performed to observe and record the position, size, and internal echo of PPLs and to preliminarily determine whether puncture biopsy could be performed.

#### 2.2.2. Conventional Ultrasound-Guided Biopsy

The appropriate position (lateral, supine, or prone position) was selected. Before the operation, an ultrasound examination was performed again to confirm the puncture path simulation design and mark the puncture point on the surface of the body. The procedure begins with a routine disinfection on the marked skin areas, followed by using 2% lidocaine for local anesthesia and finally with the installation of a sterile protective sleeve on the ultrasound probe. The puncture needle was passed through the skin along the upper edge of the rib space from the marker point to the deep chest wall, and the patient was asked to breathe. Under ultrasound guidance, the needle continued to enter the front edge of the lesion and the biopsy was completed by stimulating the biopsy gun. The tissue in the needle groove was placed on the filter paper and fixed with 10% formaldehyde solution, and then, the biopsy tissue was sent to pathological examination. In the conventional ultrasound-guided group, the active effective areas of hypoechoic, isoechoic, and hyperechoic lesions were selected as far as possible for multipoint puncture. Generally, two needles were punctured, and one needle could be added if necessary. Single puncture success rate refers to the successful puncture operation and only one puncture point (Figure 1).

#### 2.2.3. Ultrasound Contrast Method

The contrast medium was SonoVue produced in Italy, which was dissolved in 5 ml of normal saline and shaken until it became a suspension. The instrument was activated in the contrast-enhanced ultrasound mode, 2.4 ml of SonoVue microbubble suspension was rapidly injected through the cubital vein, followed by a rapid bolus of 5 ml of normal saline, and the images were observed for 5 minutes and saved. The enhancement distribution of lesions was analyzed. In the contrast-enhanced ultrasound group, the enhancement area was selected as the puncture site and the unenhanced area was avoided as far as possible. The puncture method under ultrasound guidance was the same as above, and 1-2 needles were routinely punctured (Figure 2).

### 2.3. Judgment Standard

Criteria for successful sampling were as follows: ultrasound-guided biopsy can take enough tissue for pathological diagnosis leading to successful sampling. Diagnostic criteria for malignant lesions were as follows: biopsy of effective lesions can be found in malignant cells. Criteria for the diagnosis of benign lesions were as follows: benign cells with diagnostic significance can be found in pathological tissues and this is consistent with other imaging and follow-up results. The criteria for failure of biopsy were as follows: ① The effective lesion tissues were not removed, such as necrotic tissue. ② Less-pathological tissues were removed, and pathological diagnosis was impossible. ③ The pathological tissues were removed without accurate pathological diagnosis, and the results were only pathological description. ④ The pathological diagnosis results were not consistent with those of other diagnosis results when the pathological tissue was taken out [8].

### 2.4. Statistical Analysis

SPSS 21.0 software was used for statistical analysis. The measurement data were expressed by mean ± standard deviation. The measurement data were compared between groups by the *t*-test. The counting data were compared between groups by the *x*^2^ test. *P* < 0.05 indicates that the difference between groups is statistically significant.

## 3. Results

In 110 cases, the results of surgical pathology or clinical follow-up showed that 71 cases were malignant and 39 cases were benign. Among them, we have the following.

In the conventional ultrasound group, there were 55 cases of malignant lesions, 15 cases of adenocarcinoma, 9 cases of squamous cell carcinoma, 5 cases of small cell carcinoma, 3 cases of poorly differentiated carcinoma, and 1 case of malignant mesothelioma and 22 cases of benign lesions and 14 cases of inflammatory lesions, 5 cases of inflammatory pseudotumor, 2 cases of granuloma, and 1 case of pulmonary tuberculosis.

In the contrast-enhanced ultrasound group, there were 55 cases of malignant lesions, 21 cases of adenocarcinoma, 8 cases of squamous cell carcinoma, 4 cases of small cell carcinoma, 4 cases of poorly differentiated carcinoma, and 1 case of non-small-cell carcinoma and 17 cases of benign lesions and 9 cases of inflammatory lesions, 5 cases of inflammatory pseudotumor, 2 cases of granuloma, and 1 case of pulmonary tuberculosis.

Age (*t* = 0.427, *p* = 0.67), gender (*X*^2^ = 0.367, *p* = 0.55), maximum diameter of the lesion (*t* = 1.201, *p* = 0.23), and location (*X*^2^ = 0.733) were compared between the two groups (*p* = 0.39), and the difference was not statistically significant. The success rate of single puncture in the contrast-enhanced ultrasound group (90.9%) was higher than that in the conventional ultrasound group (72.7%), and the difference was statistically significant (*p* < 0.05). The success rate of puncture in the conventional ultrasound group was 80% and that in the contrast-enhanced ultrasound group was 94.6%, and the difference was statistically significant between the two groups (*p* < 0.05). There was no significant difference in the complications of needle tract bleeding and pneumothorax after puncture between the two groups (see Table 1).

Further grouping and analysis according to the size of the lesions showed that for the cases with the largest diameter <30 mm, the difference in the single puncture success rate, the puncture success rate, and the incidence of complications (bleeding and pneumothorax) between the conventional ultrasound group and the angiography group were all different. There was no statistical significance. For the group with maximum diameter ≥30 mm, the success rate of single puncture (97.1%) and the success rate of puncture (97.1%) in the angiography-guided group were higher than those in the conventional ultrasound-guided group (70.3%, 78.4%). The difference was statistically significant (*p* < 0.05). There was no significant difference in the incidence of complications between the two groups (*p* > 0.05) (see Tables 2 and 3). In addition, there was no necrosis in the lesions in the <30 mm group; 43.1% (31/72) of the cases in the ≥30 mm group showed different degrees of necrosis during angiography.

## 4. Discussion

Lung cancer is one of the common malignant tumors, and its 5-year survival rate is only 12%–15%. Therefore, early diagnosis and timely treatment of lung cancer are particularly important [9, 10]. Peripulmonary lesions refer to the lesions below the third bronchus and above the respiratory bronchioles. Because of their proximity to the pleura, it is very difficult to puncture biopsy by using fiberoptic bronchoscopy. In view of this situation, CT and ultrasound-guided percutaneous lung biopsy can be used clinically. However, CT-guided lung biopsy has the disadvantages of large radiation dose, repeated scanning, inability to guide in real time, and high cost, so it is rarely used in clinics [11–13]. Ultrasound-guided lung biopsy has the advantages of nonradiation, real-time guidance, and economy, and ultrasound can display peripheral lung lesions near the chest wall, by which it is easy to obtain the diseased tissue. Therefore, ultrasound-guided lung biopsy is the preferred method [14–16].

Whether the effective lesion tissue can be obtained by percutaneous lung biopsy is the key to affect the diagnostic accuracy of percutaneous lung biopsy [17, 18]. Conventional ultrasound judges whether there is a necrotic area by the echo level of the lesion. It is generally believed that the extremely low-echo or echoless area is the necrotic tissue of the lesion and the low-echo, isoecho, and hyperechoic lesion area is the effective tissue. However, sometimes, the ultrasonographic images show low- to high-echo areas, and the results of puncture biopsy show the necrotic tissue. It can be seen that the echo level of the lesion cannot truly reflect whether the lesion is a necrotic tissue or an effective tissue [19, 20]. In recent years, contrast-enhanced ultrasound (CEUS) has been applied to lung examination. CEUS agents can show the blood perfusion of lesions, which is of guiding significance in puncture biopsy [21, 22]. Contrast-enhanced ultrasound is used to analyze and judge the blood perfusion of the lesion according to the enhancement of the lesion after injection of the contrast agent. The enhancement area of contrast-enhanced ultrasound is the perfusion filling area that is the active effective area, and the nonenhanced area of contrast-enhanced ultrasound is the perfusion defect or nonperfusion area that is the necrotic area, and these can guide lung biopsy in obtaining effective lesions [21, 23]. Contrast-enhanced ultrasound has some limitations; for example, the cost of contrast-enhanced ultrasound and the complexity of examination are higher than of conventional ultrasound. In addition, if contrast enhancement duration of some lesions is short, contrast-enhanced ultrasound is also prone to miss the target. Although contrast-enhanced ultrasound can show peripheral pulmonary lesions that are not close to the pleura, the interference of a certain distance between the lesion and the pleura can also easily lead to inaccurate lesion location, which leads to the failure of biopsy [24, 25].

There are significant differences in single puncture biopsy rate and puncture biopsy rate between the conventional ultrasound group and the ultrasound imaging group, which is consistent with previous research results [26, 27]. The reasons for the failure of needle biopsy were analyzed: no cancer cells were found in the biopsy results of 5 malignant lesions in the conventional ultrasound group, and the needle biopsy showed necrotic tissue, which led to the failure of needle biopsy. Among the lesions, 6 cases of biopsy failed, 5 cases were diagnosed as inflammatory lesions under the guidance of contrast-enhanced ultrasonography, and 1 case with a history of tuberculosis was found as necrotic tissue. No tumor cells were found in 3 patients in the contrast-enhanced ultrasound group, but changes in the lesions were found in subsequent follow-up, and repuncture was performed to confirm the diagnosis. There was no significant difference in the incidence of complications between the two groups (see Table 1), but it was not difficult to see that the incidence of complications in the contrast group was slightly lower than that in the conventional ultrasound group. The reason is that conventional ultrasound can show the larger blood vessels in the lesion to a certain extent, but when the blood flow velocity in the lesion is low or the patient does not cooperate, the blood flow in the lesion is not sensitive. Contrast-enhanced ultrasound can dynamically display the diameter, course, and number of blood vessels in the lesion in real time, which can avoid respiratory interference and then guide the formulation of the best puncture path to reduce the occurrence of complications [28, 29].

The success rate of puncture biopsy is affected by the size of the lesion to a certain extent [30, 31]. For larger lesions, the ultrasound image is clear, but the probability of liquefaction necrosis is higher; for smaller lesions, the ultrasound image shows poor image quality but almost no liquefaction necrosis [32, 33]. In this study, a BARD automatic biopsy gun was used for biopsy and an 18G biopsy needle was used. The needle length was 20 cm, and the ejection distance was 22 mm. When the maximum diameter of the lesion was less than 30 mm, as long as the puncture route was established, the lesion tissue could be punctured. Moreover, the probability of liquefaction necrosis in the lesion was very small, and the puncture needle could generally obtain effective tissue. When the maximum diameter of the lesion is greater than 30 mm, with the increase in the maximum diameter of the lesion, the probability of liquefaction and necrosis within the lesion also increases and the probability of the puncture needle penetrating the necrotic tissue also increases. Therefore, in this study, the influence of the diameter of the lesion on the needle biopsy was added to the comparative analysis and the lesion size of 30 mm was used as the cut-off value for further grouping [34, 35].

For the <30 mm group, there was no significant difference in puncture success rate between the conventional ultrasound group and the contrast group. The reason was that the automatic biopsy gun used in this study could obtain effective lesion tissue within the diameter range of <30 mm group. In this case, the advantages of contrast-enhanced ultrasound in locating, guiding, and distinguishing effective tissues are not obvious compared with conventional ultrasound. In addition, there was no significant difference in the incidence of complications between the two groups. For the ≥30 mm group, the success rate of single puncture and puncture in the contrast group was higher than that in the conventional ultrasound group, and the difference was statistically significant. Because there may have many new vascular tortuous and obstructions in the larger peripheral pulmonary lesions, which can easily lead to tissue ischemic necrosis. Conventional ultrasound cannot easily distinguish between the effective or necrotic tissue, while contrast-enhanced ultrasound can show the effective area of the lesion and avoid puncture to necrotic tissue, so the success rate of puncture in the contrast group is higher than that in the conventional ultrasound group [36–38]. There was no significant difference in the incidence of complications between the two groups with diameter ≥30 mm. However, the incidence of complications in these two groups was significantly lower than that in the <30 mm group. The reason was that the diameter of the lesion was large, the ultrasonographic image quality was good, the location was easy, the success rate of puncture was higher than that of the lesion with small diameter, the number of punctures were reduced, and the puncture needle was used to only puncture the lesion tissue during puncture biopsy, which would not damage the normal lung tissue around the lesion. On the other hand, the small diameter lesions are easy to be affected by respiration, it is difficult to locate, the success rate of one puncture is low, and in some cases, as long as the conditions permit, the number of punctures will be increased to obtain sufficient lesions tissue. At the same time, in some cases, the puncture needle passes through the lesion and damages the normal tissue around the lesion, which will increase the incidence of complications such as pneumothorax and bleeding to a certain extent [39].

## 5. Conclusion

For peripheral pulmonary lesions with the maximum diameter ≥30 mm, there was a significant difference in the success rate of puncture between the contrast-enhanced ultrasound group and the conventional ultrasound group and the application of contrast-enhanced ultrasound to guide puncture biopsy had better guiding significance. For peripheral pulmonary lesions with the maximum diameter <30 mm, there was no significant difference in the puncture success rate between the contrast-enhanced ultrasound group and the conventional ultrasound group. Due to the small sample size of this study, it is necessary to expand the sample for further discussion.

## Figures and Tables

**Figure 1:** A patient in the conventional ultrasound group, male, 56 years old. (a) Ultrasonography showed a hypoechoic mass in the middle lobe of the right lung, with a size of 51 mm∗38 mm, and the echo was still uniform. (b) Color Doppler displayed a little blood flow signal. (c) The needle was passed through the pleura, into the lesion, and cut for biopsy. (d) Five minutes after needle extraction, no obvious bleeding and pneumothorax and other complications were found.

**Figure 2:** A patient in the contrast-enhanced ultrasound group. (a) Ultrasound examination showed a hypoechoic mass in the lower left lung, 43 mm ∗40 mm in size, with an uneven echo. (b) After injection of the contrast agent, it showed uneven enhancement. (c) The puncture needle was passed through the pleura, into the lesion, and cut for biopsy. (d) Five minutes after needle extraction, no obvious bleeding and pneumothorax and other complications were found.

**Table 1:** Basic information of the conventional ultrasound group and contrast-enhanced ultrasound group.

Group	Age	Maximum diameter	Location (lung)		Sexuality	
			Upper middle lobe	Lower lobe	Male	Female
Conventional ultrasound group	68.7 ± 14.0	45.4 ± 22.4	38	17	35	20
Contrast-enhanced ultrasound group	67.8 ± 13.3	51.0 ± 26.5	42	13	38	17
c^2^ value/*t* value	0.427	1.201	0.733	0.367		
*p* value	0.67	0.23	0.39	0.55		

Group	Success rate of single puncture	Success rate of puncture	Pneumothorax rate			
Conventional ultrasound group	72.7% (40/55)	80.0% (44/55)	16.4% (9/55)			
Contrast-enhanced ultrasound group	90.9% (50/55)	94.6% (52/55)	10.9% (6/55)			
*X* ^2^ value/*t* value	6.111	4.01	0.695			
*p* value	0.013	0.045	0.405			

**Table 2:** Related indicators of biopsy for the <30 mm group.

Group	Success rate of single puncture	Success rate of puncture	Needle bleeding rate	Pneumothorax rate
Conventional ultrasound group	77.8% (14/18)	83.3% (15/18)	27.8% (5/18)	27.8% (5/18)
Contrast-enhanced ultrasound group	80.0% (16/20)	90.0% (18/20)	25.0% (5/20)	20.0% (4/20)
*X* ^2^ value/*t* value	0.027	0.016	0.037	0.309
*p* value	0.869	0.899	0.848	0.578

**Table 3:** Related indicators of biopsy for the ≥30 mm group.

Group	Success rate of single puncture	Success rate of puncture	Needle bleeding rate	Pneumothorax rate
Conventional ultrasound group	70.3% (26/37)	78.4% (29/37)	10.8% (4/37)	10.8% (4/37)
Contrast-enhanced ultrasound group	97.1% (34/35)	97.1% (34/35)	2.9% (1/35)	5.7% (2/35)
*X* ^2^ value/*t* value	7.517	4.202	0.745	0.126
*P* value	0.006	0.04	0.388	0.722

## Data Availability

No data were used to support this study.

## References

[1] Tang M., Song J. Q., Zheng X. X. (2020). etc. Contrast analysis of contrast-enhanced ultrasonography and conventional ultrasound-guided puncture for peripheral pulmonary lesions. *Chinese Journal of Ultrasound in Medicine*.

[2] Yang P.-C. (1997). Ultrasound-guided transthoracic biopsy of peripheral lung, pleural, and chest-wall lesions. *Journal of Thoracic Imaging*.

[3] Sperandeo M., Dimitri L., Pirri C., Trovato F. M., Catalano D., Trovato G. M. (2014). Advantages of thoracic ultrasound-guided fine-needle aspiration biopsy in lung cancer and mesothelioma. *Chest*.

[4] Dong Y., Mao F., Wang W.-P., Ji Z.-B., Fan P.-L. (2015). Value of contrast-enhanced ultrasound in guidance of percutaneous biopsy in peripheral pulmonary lesions. *BioMed Research International*.

[5] Li Q., Nie F., Yang D., Li J. (2017). Application of contrast enhanced ultrasound combined biopsy in qualitative diagnosis of peripheraI pulmonary lesions. *Chinese Journal of Interventional Imaging and Therapy*.

[6] Gorg C., Bert T., Gorg K. (2005). Contrast-enhanced sonography for differentiaI diagnosis of pleurisy and focal pIeural lesions of unknown cause. *Chest*.

[7] Hong-Xia Z., Wen H., Ling-Gang C. (2016). A new method for discriminating between bronchial and pulmonary arterial phases using contrast-enhanced ultrasound. *Ultrasound in Medicine & Biology*.

[8] Yang R. Y., Ng D., Jaskolka J. D., Rogalla P., Sreeharsha B. (2014). Evaluation of percutaneous ultrasound—guided biopsies of solid mass lesions of the pancreas: a center’s 10-year experience. *Clinical Imaging*.

[9] Detterbeck F. C., Franklin W. A., Nicholson A. G. (2016). The IASLC lung cancer staging project: background data and proposed criteria to distinguish separate primary lung cancers from metastatic foci in patients with two lung tumors in the forthcoming eighth edition of the TNM classification for lung cancer. *Journal of Thoracic Oncology*.

[10] Zeng C., Wen W., Morgans A. K., Pao W., Shu X.-O., Zheng W. (2015). Disparities by race, age, and sex in the improvement of survival for major cancers: results from the national cancer institute surveillance, epidemiology, and end results (SEER) program in the United States, 1990 to 20l0. *JAMA Oncology*.

[11] Sehgal I. S., Dh00Ria S., Bal A. (2019). A retrospective study comparing the ultrathin versus conventional bronchoscope for performing radial endobronchial ultrasound in the evaluation of peripheral pulmonary lesions. *Lung India : Official Organ of Indian Chest Society. Lung*.

[12] Gupta A., Suri J. C., Bhattacharya D. (2018). Comparison of diagnostic yield and safety profile of radial endobronchial ultrasound-guided bronchoscopic lung biopsy with computed tomography-guided percutaneous needle biopsy in evaluation of peripheral pulmonary lesions: a randomized controlled trial. *Lung India*.

[13] Ko J. P., Shepard J. O., Drucker E. A. (2001). Factors influencing pneumothorax rate at 1ung biopsy: are dweIl time and angIe of pleural puncture contributing factors?. *Radiology*.

[14] Yamamoto N., Watanabe T., Yamada K. (2019). Efficacy and safety of ultrasound (US)guided percutaneous needle biopsy for peripheral 1ung or pleural lesion: comparison with computed tomography (CT)guided needle biopsy. *Journal of Thoracic Disease*.

[15] Chavez C., Sasada S., Izum0 T. (2015). Endobronchial u1trasound with a guide sheath for small malignant pulmonary nodules: a retrospective comparison between central and peripheral locations. *Journal of Thoracic Disease*.

[16] Cao B. S., Wu J. H., Li X. L., Liao G.-Q. (2011). Sonographically guided transthoracic biopsy of peripheral lung and mediastinal 1esions: roie of contrast—enhanced sonography. *Ultrasound Med*.

[17] Hsu W. H., Chiang C. D., Hsu J. Y., Kwan P. C., Chen C. L., Chen C. Y. (1996). Ultrasound-guided fine needle aspiration biopsy of lung cancers. *Journal of Clinical Ultrasound*.

[18] Wu W., Chen M. H., Yin S. S. (2006). The role of contrast-enhanced sonography of focal liver lesions before percutaneous biopsy. *American Journal of Roentgenology*.

[19] Caturelli E., Biasini E., Bartolucci F. (2002). Diagnosis of hepatocellular carcinoma complicating liver cirrhosis :utility of repeat ultrasoundguided biopsy after unsuccessful first sampling. *CardioVascular and Interventional Radiology*.

[20] He W., Hu X. D., Wu D. f. (2006). Ultrasonography-guided percutaneous microwave ablation of peripheral lung cancer. *Clinical Imaging*.

[21] Caremani M., Benci A., Lapini L. (2008). Contrast enhanced ultrasonography (CEUS) in peripheral lung lesions: a study of 60 cases. *Journal of Ultrasound*.

[22] Zheng Y. L., Yin X. Y., Xie X. Y. (2010). Value of contrast-enhanced ultrasonography in assessing the vascularity of liver metastases: comparison with contrast-enhanced computed tomography. *Journal of Ultrasound in Medicine*.

[23] Yi D., Feng M., Wenping W., Ji Z.-B., Fan P.-L. (2015). Value of contrast-enhanced ultrasound in guidance of percutaneous biopsy in peripheral pulmonary lesions. *BioMed Research International*.

[24] Guo Y. Q., Liao X. H., Li Z. X. (2018). Ultrasound—guided percutaneous needle biopsy for peripheral pulmonary lesions: diagnostic accuracy and influencing factors (Article). *Ultrasound in Medicine and Biology*.

[25] Wang S., Yang W., Zhang H., Xu Q., Yan K. (2015). The role of contrast-enhanced ultrasound in selection indication and improving diagnosis for transthoracic biopsy in peripheral pulmonary and mediastinal lesions. *BioMed Research International*.

[26] Chen B. L., Huang P. T., Ye F., Chen L.-M. (2012). The value of contrast-enhanced ultrasonography in differential diagnosis of peripheral lung cancer. *Chinese Journal of Ultrasound in Medicine*.

[27] Yang H. H., Liu J. J., Tang X. H., Li Z.-X. (2014). Analysis of factors affecting the accuracy of ultrasound-guided peri-pulmonary biopsy. *Chinese Journal of Medical Imaging*.

[28] Sartori S., Postorivo S., Vece F. D., Ermili F., Tassinari D., Tombesi P. (2013). Contrast-enhanced ultrasonography in peripheral lung consolidations: what’s its actual role?. *World Journal of Radiology*.

[29] Eldridge L., Moldobaeva A., Zhong Q. (2016). Bronchial artery angiogenesis drives lung tumor growth. *Cancer Research*.

[30] Fang Q., Huang W. J., Qiu Y. D., Peng W.-W. (2017). Ultrasound-guided biopsy of peripheral pulmonary lesions on the diagnosis rate and influencing factors of complications. *Chinese Journal of Ultrasound in Medicine*.

[31] Tsukada H., Satou T., Iwashima A., Souma T. (20oo). Diagnostic accuracy of CT guided automated needle biopsy of lung nodules. *American Journal of Roentgenology*.

[32] Liao W. Y., Chen M. Z., Chang Y. L. (2000). US-guided transthoracic cutting biopsy for peripheral thoracic lesions less than 3 cm in diameter. *Radiology*.

[33] Gorg C., Kring R., Bert T. (2006). Transcutaneous contrast-enhanced sonography of peripheral lung lesions. *American Journal of Roentgenology*.

[34] Yeow K. M., Tsay P. K., Cheung Y. C., Lui K. W., Pan K. T., Chou A. S. B. (2003). Factors affecting diagnostic accuracy of CT-guided coaxial cutting needle lung biopsy: retrospective analysis of 631 procedures. *Journal of Vascular and Interventional Radiology*.

[35] Arakawa H., Nakajima Y., Kurihara Y., Niimi H., Ishikawa T. (1996). CT-guided transthoracic needle biopsy: a comparison between automated biopsy gun and fine needle aspiration. *Clinical Radiology*.

[36] Jing K., Jingjing F., Wei Y. (2020). Contrast-enhanced ultrasound features of mediastinal lymphomas and thymic epithelial tumors. *Journal of Clinical Ultrasound*.

[37] Chen M. H., Yan K., Sun X. M. (2001). Diagnostic value of ultrasound-guided needle biopsy for central lung tumors. *Chinese Journal of Ultrasound in Medicine*.

[38] He W., Cheng Y., Zhang H. X. (2011). etc. Clinical application of percutaneous biopsy of peripheral lung tumors guided by contrast-enhanced ultrasound. *Chinese Journal of Ultrasound in Medicine*.

[39] Scisca C., Rizzo M., Maisano R. (2002). The role of ultrasound-guided aspiration biopsy of peripheral pulmonary nodules: our experience. *Anticancer Research*.

